# Melanin pigment of *Streptomyces puniceus* RHPR9 exhibits antibacterial, antioxidant and anticancer activities

**DOI:** 10.1371/journal.pone.0266676

**Published:** 2022-04-25

**Authors:** Ravinder Polapally, Manasa Mansani, Karthik Rajkumar, Sandeepta Burgula, Bee Hameeda, Alaa Alhazmi, Farkad Bantun, Atiah H. Almalki, Shafiul Haque, Hesham Ali El Enshasy, R. Z. Sayyed

**Affiliations:** 1 Department of Microbiology, University College of Science, Osmania University, Hyderabad, India; 2 Medical Laboratory Technology Department, Jazan University, Jazan, Saudi Arabia; 3 SMIRES for Consultation in Specialized Medical Laboratories, Jazan University, Jazan, Saudi Arabia; 4 Department of Microbiology, Faculty of Medicine, Umm Al-Qura University, Mecca, Saudi Arabia; 5 Department of Pharmaceutical Chemistry, College of Pharmacy, Taif University, Taif, Saudi Arabia; 6 Addiction and Neuroscience Research Unit, College of Pharmacy, Taif University, Al-Hawiah, Taif, Saudi Arabia; 7 Research and Scientific Studies Unit, College of Nursing and Allied Health Sciences, Jazan University, Jazan, Saudi Arabia; 8 Bursa Uludağ University Faculty of Medicine, Görükle Campus, Nilüfer, Bursa, Turkey; 9 Institute of Bioproduct Development (IBD), Universiti Teknologi Malaysia (UTM), Skudai, Johor Bahru, Johor, Malaysia; 10 School of Chemical and Energy Engineering, Faculty of Engineering, Universiti Teknologi Malaysia (UTM), Skudai, Johor Bahru, Johor, Malaysia; 11 City of Scientific Research and Technology Applications (SRTA), New Burg Al Arab, Alexandria, Egypt; 12 Department of Microbiology, PSGVP Mandal’s Arts, Science, and Commerce College, Shahada, India; PMAS Arid Agriculture University: University of Arid Agriculture, PAKISTAN

## Abstract

The present study reveals the production of dark, extracellular melanin pigment (386 mg/L) on peptone yeast extract iron agar medium by *Streptomyces puniceus* RHPR9 using the gravimetric method. UV-Visible, Fourier Transform Infrared (FTIR), and Nuclear Magnetic Resonance (^1^H) (NMR) spectroscopy confirmed the presence of melanin. Extracted melanin showed antibacterial activity against human pathogens such as *Bacillus cereus*, *Staphylococcus aureus*, *Pseudomonas aeruginosa*, and *Escherichia coli* except for *Klebsiella pneumoniae*. A potent free radical scavenging activity was observed at 100 μg/mL of melanin by the DPPH method with a concentration of 89.01±0.05% compared with ascorbic acid 96.16±0.01%. Antitumor activity of melanin was evaluated by MTT assay against HEK 293, HeLa, and SK-MEL-28 cell lines with IC_50_ values of 64.11±0.00, 14.43±0.02, and 13.31±0.01 μg/mL respectively. Melanin showed maximum anti-inflammatory activity with human red blood cells (hRBC) (78.63 ± 0.01%) and minimum hemolysis of 21.37±0.2%. The wound healing potential of the pigment was confirmed on HeLa cells, cell migration was calculated, and it was observed that cell migration efficiency decreased with an increase in the concentration of melanin. To our knowledge, this is the first evidence of melanin produced from *S*. *puniceus* RHPR9 that exhibited profound scavenging, anti-inflammatory and cytotoxic activities.

## Introduction

Interest in microbially derived pigments has gained significance for quite a long time due to toxic effects caused by their synthetic counterparts [1]. This is due to their higher stability, availability, easy harvestability and yield [2]. In nature, the colored pigments produced by microorganisms like algae, bacteria, fungi, yeasts, and protozoa have considerable advantages over synthetic or inorganic colors [3]. Microbial pigments are non-toxic, non-carcinogenic, and biodegradable with many industrial applications [4]. Microorganisms produce various pigmented byproducts like bacteriochlorophylls, carotenoids, flavins, indigoids, melanin, monastic, phenazine, astaxanthin, and ß carotene [4]. A broad variety of cell-specific biological activities have been reported by many of these compounds and their derivatives at active/inhibitory/lethal/sub-lethal concentrations i.e., Effective Dose (ED), Growth Inhibition Concentration (GIC), Minimum Inhibitory Concentration (MIC), and half-full Effectiveness Concentration (EC_50_) [5].

Production of melanin from microorganisms has been an environmentally friendly approach and economical alternative to the chemical synthesis of melanin [6]. Melanins are available in different forms, such as eumelanin, pheomelanin, and allomelanins [7]. The black-brown colored pigment of eumelanin formed due to the oxidative polymerization of tyrosine or phenylalanine to L-DOPA is further transformed into melanin [8, 9]. Streptomyces are widely used for producing secondary metabolites (antibiotics, enzymes, antitumor, striking pigments, antioxidants) in biotechnology as antioxidant, anti-inflammatory and antimicrobial [10]. They can be used in the food and pharma sector [11]. Pigments produced by microorganisms are preferred over plant-based pigments as environmental factors do not interfere in their production [12]. Melanin is commonly used in the drug preparation, pharmacology, textile, agricultural, cosmetic, and food processing industries [13, 14]. Melanin plays an important role in microorganisms overcoming thermal, chemical, and biochemical stress conditions [15]. Melanin influences humans’ skin color and plays a significant role in protection against UV radiation. Water-soluble melanin is widely used in sunscreens, solid plastic films, lenses, lacquer paints, and other formulations to provide greater protection from UV [16]. Significant biological activities of melanin include protection to liver [17] antibacterial [18] antitumor [19] antioxidant [20] and anti-inflammatory [21]. The present study was aimed to extract melanin produced from *Streptomyces puniceus* RHPR9. isolated from the rhizosphere of medicinal plant (*Coscinium fenestratum*). Extracted melanin was characterized by UV-visible absorption spectrometry, Fourier-Transform Infrared Spectroscopy (FTIR), and Nuclear Magnetic Resonance (NMR). The pigment thus obtained from *S*. *puniceus* RHPR9 was tested for antibacterial, antioxidant, antitumor, anti-inflammatory and wound healing properties.

## Materials and methods

*Streptomyces* sp. was isolated from the rhizosphere of the medicinal plant (*Coscinium fenestratum*) from the Western Ghats of Karnataka, India (Ravinder et al. published elsewhere). Actively growing culture of *S*. *puniceus* RHPR9 was inoculated as a spot at the center of Petri plate and incubated at 30 °C for seven days. Pigment production was observed at regular intervals every 24 h for one week. The Brown to the black coloration of diffused pigment around the colony indicates melanin production.

### Media used for pigment production by *S*. *puniceus* RHPR9

The production of melanin pigment was checked on different synthetic media such as Peptone Yeast Extract Iron Agar (PYIA), Tyrosine Agar (TA), Glycerol Peptone Agar (GPE), and Starch Casein Agar (SCA). Among all media, the PYIA medium was suitable for producing melanin, and hence it was used for further studies. The single isolated colony of *S*. *puniceus* RHPR9 was inoculated in an Erlenmeyer flask (250 mL) that consisted of 100 mL PYI broth medium and incubated for 30 °C and 150 rpm for seven days [22]. This was used as a seed medium for further studies.

### Inoculum preparation and growth conditions for melanin production of *S*. *puniceus* RHPR9

*S*. *puniceus* cultured inoculum (1%) was grown in 250 mL PYI broth medium (pH 6.7) for seven days on a rotatory orbital shaker (150 rpm) at 30 °C. Following incubation, the broth was centrifuged at 10,000 rpm for 10 min, and supernatant was subjected to tyrosinase assay to determine melanin activity [23].

### Extraction, estimation, and purification of melanin pigment

The tyrosinase assay was used to check the breakdown of extracellular black/brown pigment. Tyrosinase assay was performed to measure the amount of melanin produced by *S*. *puniceus*. The assay consisted of 2 mL of cell-free supernatant, 2 mL of 0.1 M phosphate buffer (pH 7), and 1 mL of 10 mM tyrosine solution. The reaction mixture was incubated for 15 min at 37 °C, and red color formed due to dopachromes was estimated at 480 nm using UV–Visible spectrophotometer [24].

Melanin was extracted from fermentation broth by removing cell debris using a centrifuge at 5000 rpm at room temperature for 15 min. The pH of the supernatant was set to 3 to precipitate melanin. Precipitated melanin was further dissolved in 6 M HCl for 4 h for digestion of bounded protein followed by centrifugation at 5000 rpm for 15 min. Extracted melanin was washed several times with sterilized water and then centrifugated for 15 min at 10,000 rpm [18, 25, 26].

### Characterization of pigment by physiochemical methods

#### Spectroscopic examination of extracted melanin pigment

Extracted melanin pigment obtained above was dissolved in 0.5 M NaOH solution and then analyzed in UV-visible (near-infrared wavelengths of 200–800 nm) spectrophotometer and NaOH (0.5 M) solution was used as blank [20, 24].

#### Fourier transform infrared spectroscopy

Extracted melanin and KBr pellets were mixed in mortar and ground to mix lumps of melanin and KBr into a fine film. This was scanned in FTIR spectrophotometer at 4000–400 cm^-1^ [15].

#### ^1^H NMR spectroscopic studies of melanin pigment

Melanin pigment was subjected to further analysis using a nuclear magnetic resonance spectrometer (NMR). The ^1^H NMR spectrum was measured at 25 °C using a BRUKER Spectrometer equipped with a triple-resonance (^1^H, _13_C, _15_N) inverse probe (5 mm in diameter) that contained 600 μL of the sample, with deuterated chloroform as a solvent [27].

### Bioassays of melanin pigment

#### Antibacterial activity

Extracted crude melanin was dissolved in 1M NaOH and tested for antibacterial activity by agar well method against *Bacillus cereus* MTCC492, *Staphylococcus aureus* MTCC6538, *Pseudomonas aeruginosa* MTCC741, *Klebsiella pneumonia* MTCC432, and *Escherichia coli* MTCC1304. Crude melanin pigment (@different aliquots) 31.25 to 250 μg/mL was loaded in agar wells, and plates were incubated at 37 °C for 24 h and observed for a zone of inhibition [19].

#### Antioxidant activity

Free radicals-scavenging behavior was calculated by the DPPH (1, 1, 1 diphenyl-2-picryl hydroxyl) method. A 80 μL of DPPH solution (0.2mg/mL) in methanol and 20 μL of different concentrations (20 to 100 μg/mL) of melanin pigment was dissolved in methanol and added to each well of the microplate. Ascorbic acid was used as standard. The mixture was vigorously shaken and kept in the dark for 30 min at room temperature. Freshly processed 40 μg/mL DPPH (2 mL) in methanol was added to each tube that contained different concentrations of pigment (20 to100 μg/mL) and standard (1mg/1mL), followed by vigorous stirring and allowed to stand in a dark place for 30 min. The tube without pigment was maintained as control, and methanol was used as blank. Then the reaction mixture was measured at 517 nm, and the following formula was used to calculate [28].


$$\text{\%}\;\text{Radical}\;\text{scavenging}\;\text{activity}=\frac{\text{Control}\;\text{O}.\text{D}-\text{Test}\;\text{O}.\text{D}}{\text{Control}\;\text{O}.\text{D}}\text{X}100$$

#### Anticancer activity

Cytotoxicity of the pigment was evaluated on cell lines, i.e. Human embryonic kidney 293 (HEK), Human cervical cancer (HeLa), and SK-MEL-28 using MTT (3-(4, 5-dimethylthiazol-2-yl)-2, 5-diphenyl tetrazolium bromide) assay according to the method defined by Zhnag et al. [41]. Cells were obtained from the National Center for Cell Science (NCCS), Pune, India and maintained in Minimum Essential Medium (MEM) with 10% fetal bovine serum (FBS) in a humidified 5% CO_2_ incubator. Log phase cells were harvested using Trypsin-EDTA solution, washed with PBS, and suspended in 20 mL of MEM. Cells were seeded at a final concentration of 3 x 10^4^ cells/200μL/well in flat-bottom 96-well microplates incubated at 37 °C, 5% CO_2_, and 95 percent relative humidity for 24 h. After which, cells were serum-starved overnight and treated with pigment dissolved in dimethyl sulfoxide(DMSO) at concentrations of 0.5, 1, 2, 5, 10, 25, 50, 75, and 100 μg/mL in triplicates for 24 h. Later, the media was replaced by 5 mg/mL MTT dissolved in PBS and incubated at 37 °C for 4 h after which the MTT dye was removed and DMSO was added followed by measurement of O.D at 595 nm [29].

#### Anti-inflammatory activity

*In vitro* Human Red Blood Cells (hRBC) membrane stabilization method was used to determine the anti-inflammatory activity of melanin pigment. Blood samples were collected from human volunteers and combined with the same volume of Alsever’s solution (0.8% sodium citrate, 0.42% sodium chloride, 0.5% citric acid, and 2% dextrose in water), centrifuged at 3000 rpm. The pellet was washed with saline (0.85% NaCl, pH 7.4), and then 10% suspension was made with saline; 0.5 mL of this hRBC solution was added to 2 mL of melanin pigment (different concentrations; 62.5, 125, 250, 500 μg/mL) and 1 mL of phosphate buffer (0.15 M, pH 7.4). The same quantity of synthetic test medication (Diclofenac) per 1 mL of hRBC solution was used as a reference drug and different amounts of the pigment i.e. 62.5, 125, 250, and 500 μg/mL. All samples were incubated for 30 min at 37 °C and centrifuged. Hemoglobin content in the supernatant fluid was estimated using a UV spectrophotometer at 560 nm. Percentage inhibition of hemolysis was determined by the following equation [30].


$$\text{Hemolysis}\;\text{inhibition}\;\left(\text{\%}\right)=\frac{\text{OD}\;\text{of}\;\text{control}-\text{OD}\;\text{of}\;\text{test}\;\text{sample}}{\text{OD}\;\text{of}\;\text{Control}}\text{x}100$$

$$\text{Percentage}\;\text{of}\;\text{protection}=100-\frac{\text{OD}\;\text{of}\;\text{Test}}{\text{OD}\;\text{of}\;\text{Control}}\text{x}100$$

#### Cell migration assay

A cell migration assay determined the wound healing property of melanin. HeLa cells were seeded 3x10^5^ cells/well into a 6 well plate (Nunc, Denmark) and allowed to grow for 24 h to get a monolayer with a 70–80% confluency. After 24 h, the monolayer was scratched gently using a sterilized 100 μL pipette tip, and the scratch was performed in the form of a cross in each well. Cells were washed twice with Dulbecco’s PBS. Later, a fresh medium that contained the pigment was added at various concentrations (0.5–10 μg/mL) in the wells, and the cells were allowed to grow for 24 h. Images were obtained from the same field immediately after scratching and 24 h. The total width of the wound area was calculated by using ImageJ software. Untreated scratched cells were taken as controls, and the percentage of wound closure was calculated using the following formula [31].


$$\text{Wound}\;\text{closure}\;\left(\text{\%}\right)=\frac{\text{Wound}\;\text{area}\;\text{at}\;0\;\text{h}–\text{Wound}\;\text{area}\;\text{at}\;24\text{h}}{\text{Wound}\;\text{area}\;\text{at}\;0\;\text{h}}\text{x}\;100$$

## Results

### Production of melanin pigment using PYI broth medium

*Streptomyces puniceus* RHPR9 isolated from the rhizosphere of medicinal plant (*C*. *fenestratum*) in the Western Ghats of Karnataka, India, produced copious amounts of melanin pigment. The development of brown or black color on PYIA medium around colonies of *Streptomyces puniceus* RHPR9 indicated melanin production (Fig 1A). Among the various media used for melanin production, isolate *Streptomyces puniceus* RHPR9 produced maximum melanin in the PYIA medium (Fig 1B).

**Fig 1:** A) Melanin pigment on peptone yeast extract iron agar medium by *S*. *puniceus* RHPR9. B). Production of melanin pigment on peptone yeast extract iron broth medium by *S*. *puniceus* RHPR9. C). Crystalline form of melanin pigment from *S*. *puniceus* RHPR9.

### Extraction, estimation, and purification of melanin pigment

Purified melanin has pure black colour, which is characteristic among all melanins. Among all the different media used to produce melanin pigment (Fig 1C), the PYI broth medium showed a maximum yield of 386 mg dry wt/L gravimetrically and tyrosinase activity was 640 μg/mL.

### Characterization of pigment by physiochemical methods

#### Spectroscopic examination of extracted melanin pigment

The UV-visible absorption spectrum of the extracted melanin at 200–800 nm showed maximum absorption of melanin pigment at 250 nm in the UV region, which declined and indicated the characteristic property of melanin pigment (Fig 2).

**Fig 2:** UV-visible absorbance spectrum of purified melanin pigment of *S*. *puniceus* RHPR9.

#### Fourier transform infrared spectroscopy

FTIR spectrum of melanin revealed a peak of about 3421.83 and 3443 cm^−1^, similar to the O-H group, a small band of 2956.97 cm^−1^ could be attributed to stretch signals of the aliphatic C-H group. Vibration in 3600–2800 cm^−1^ region due to O-H and N-H indicates amine, amide, or carboxylic acid, phenolic and aromatic in both indolic and pyrrolic systems. The secondary N-H unit bending is associated with a peak observed close to 1629.90 cm^−1^. The broad distinctive band around 1650–1620 cm^−1^ (1629.90 cm^−1^) is assigned to aromatic ring vibrations C = C of amide IC = O and/or COO groups. The peak of N-H stretch vibration at 1546.96 cm^−1^ specifies that pigment has a distinctive melanin indole structure. Phenolic C-OH stretch at 1246.06 cm^−1^ corresponds to phenolic compounds. The maximum focus at 1051.24 cm^−1^ indicates C-H in the plane of an aliphatic structure representative of melanin pigment. The peak detected at 835.21 cm^−1^ is due to aromatic group C-H, and weak bands below 700 cm^−1^ represent the alkene C-H replacement in melanin (Fig 3). Based on UV-Visible absorption and FTIR data, the pigment produced from *S*. *puniceus* RHPR9 was concluded as eumelanin.

**Fig 3:** FTIR spectrum of melanin pigment of *S*. *puniceus* RHPR9.

#### ^1^H NMR spectroscopic studies of melanin pigment

^1^H NMR spectrum of the obtained melanin pigment from *S*. *puniceus* RHPR9 exhibited vibrations in the range of 8.3 to 6.0, the strong aromatic resonances assigned to melanin polymer indole or pyrrole repeated groups. Absorption peaks at 0.973 to 4.282 ppm (parts per million) are assigned for protons attached to methyl or methylene groups attached to nitrogen and/or oxygen atoms. The absorption peak at 2.1 ppm is recognized as C_14_-H and C_23_-H of melanin. Vibrations between 1.0 and 3.00 ppm may be allocated to the existence of an indole-linked NH-group. Vibration at 0.9 ppm correlates to an aliphatic methyl group (Fig 4).

**Fig 4:** ^1^HNMR Spectroscopy of the melanin pigment of *S*. *puniceus* RHPR9.

### Bioassays of melanin pigment

#### Antibacterial activity

Antibacterial activity of melanin pigment was evaluated by agar well method. Melanin pigment exhibited antibacterial activity against Gram-positive and Gram-negative bacteria at concentrations of 31.25 to 250 μg/mL. Test microorganisms include *B*. *cereus* MTCC492, *S*. *aureus* MTCC6538, *P*. *aeruginosa* MTCC741, *K*. *pneumonia* MTCC432, and *E*.*coli* MTCC1304. The highest concentration of melanin pigment (250 μg/mL) showed inhibition against *B*. *cereus* with a zone size of 25 mm and *K*. *pneumoniae* (12 mm).

#### Antioxidant activity

DPPH method was used to check the ability of melanin to scavenge free radicals to assess its antioxidant activity. Melanin pigment exhibited strong antioxidant activity of 89.01±0.02% at 100 μg/mL concentration compared to 96.16±0.01% activity with the same amount of ascorbic acid.

#### Anticancer activity

Further, the extracted melanin pigment was evaluated for its anticancer properties on HEK 293, HeLa, and SK-MEL-28 by MTT assay. Percentage of cell viability monitored after 24 h was 53.59±0.11, 51.85±0.01, and 17.7±0.1 for HEK 293, HeLa, and SK-MEL-28, respectively, when 100 μg/mL melanin was used. Maximum IC_50_ value (μg/mL) of 14.43 ±0.02 with HeLa cells, 13.31±0.01 with SK-MEL-28, and 64.11±0.00 with HEK 293 (Fig 5).

**Fig 5:** Cell viability assays of HEK 293, HeLa, and SK-MEL-28 cell lines were tested for 24 h with various concentrations ranging from 0.5 to 100 μg/mL in 96 well plates. The cell viability was determined at maximum absorption at 570 nm. A graph was depicted with melanin concentrations on the x-axis and percent viable cells on the y-axis.

#### Anti-inflammatory activity

Melanin provided maximum protection (78.63 ± 0.01) and minimum hemolysis (21.37±0.2%) when tested for *in vitro* anti-inflammatory activity at a dose of 500 μg/mL. The results were correlated to that of standard drug, i.e., Diclofenac at similar concentrations protected in a range of (80.76 ±0.01 and 19.24±0.1%) the cells tested (Fig 6).

**Fig 6:** In-vitro wound-healing assay on HeLa cells: (0 h) wound was made by scratching a monolayer of HeLa cells with 100 μl sterile tip and treated with indicated concentrations of melanin. To assess the degree of wound healing, cell migration towards the scratched areas was visualized and photographed at 0 h and then at 24 h.

#### Cell migration assay

Melanin had a significant effect on HeLa cell line migration patterns. Cell migration was significantly reduced at higher concentrations of melanin treatment, as observed in wound healing assay. The percentage of cells that invade the wounded areas was reduced in melanin (10 μg/mL) treated HeLa with reduced cell proliferation (Fig 7).

**Fig 7:** The data was calculated from two independent where random fields were selected and quantified using ImageJ software.

## Discussion

Medicinal plants and their products have been used in traditional medicine for ages. They serve as a source of a wide range of bioactive molecules like antibiotic, antiviral, and antifungals. These compounds are often of plant origin, but microbiota associated with these medicinal plants also exhibit such diversified properties [32]. Recently, an endophyte related to this plant, *Enterobacter* spp., was known to inhibit biofilm formation [33]. Actinobacteria isolated from varied sources are reported for secondary metabolites production with different applications [34]. In this study, strain RHPR9 produced maximum melanin (386 mg/L) in PYI broth medium strain vis-a-vis low amount (350 mg/L) of melanin produced by *Streptomyces glaucescens* strain NEAE-H [15] and yeast melanin by *Yarrowia lipolytica* was 160 mg/L in M8 medium [35].

Melanin polymers are the structural components of melanin granules. The development of granules and their size are significantly influenced by pH. A low pH promotes aggregate growth and a high pH, causing the granules to break up into tiny particle-oligomers with a reduced degree of polymerization. The maximum absorption of melanin concentration was detected at 250 nm in the UV region by strain RHPR9. The usual range of melanins absorption was 200–250 nm [36]. Similar findings were reported on the absorption spectrum of melanin obtained from *Phyllosticta capitalensis* [37]. Melanin absorption peak of *Streptomyces glaucescens* NEAE-H [15] was in the range of 250 nm, *Chroogomphus rutilus* (mushroom), was at 212 nm [9] and yeast (*Cryptococcus rajasthanensis*) at 244 nm [38].

FTIR spectra of melanin (Fig 3) revealed a peak of 3421.83 cm^−1^, similar to the OH group, a small band of 2956.97 cm^−1,^ which can be attributed to stretch signals of the aliphatic C-H group. Previous studies revealed the distinctive bands around 1650–1620 cm^−1^ indicate melanin pigment, and in this study, the band at 1629.90 cm^−1^ was observed. Peaks at 1211.34 to 1383.01 cm^−1^ correspond to synthetic melanin’s anhydrides (C-O) class and all bacterial pigments extracted [32–40]. ^1^H NMR spectral data revealed melanin pigment production in strain RHPR9 (Fig 4). The comparable absorption spectra have been recorded for fungal melanin obtained by *Auricularia auricular* [41] and *Cryptococcus rajasthanensis* [38].

Antibacterial activity of extracted melanin pigment from strain RHPR9 was maximum against *B*. *cereus* and minimum with *K*. *pneumoniae* Table 1. Similar findings were reported by Soundra et al. [42], with black yeast (*Hortaea werneckii*) melanin pigment, which showed a maximum zone of inhibition against *Salmonella typhi* (17 mm) and a minimum for *K*. *pneumoniae* (11 mm). Avilla et al. [38] reported the antibacterial activity of melanin against Gram-positive bacterium, *Bacillus subtilis*, and Gram-negative bacterium, *Pseudomonas aeruginosa*. This might be due to the difference in the structure of cell wall of gram positive and gram negative bacteria. It can be attributed to the reactive oxygen species produced by melanin that cause cell death by damaging the structure and function of cellular proteins and other components. A similar study of antibacterial and antioxidant activities of melanin obtained from *Equus ferus* hair against was reported by Tahmineh Rahmani Eliato [43]. Significant antioxidant activity (89% by DPPH method) was exhibited by melanin pigment characterized in this study. Previous studies have shown that increased melanin levels have increased antioxidant activity. However, the free radical scavenging activity varied from 56.58 to 68.91% [28] and 87–96% [44]. The free radicals and other reactive species are easily scooped up by melanin pigment due to valence electrons in their molecules. They are used as antioxidants to facilitate their use in cosmetic products, which reduces tissue damage due to toxins [20]. Melanin acts as a potent anticancer agent that kills the cancer cells with low concentrations without causing damage to normal cells. Table 1 depicts the significant anticancer activity of melanin in this study. According to previous reports, IC50 values with a range of 1–10, 11–20, 21–50, and 51–100 are graded as very strong, strong, moderate, and weak cytotoxicity activity. The melanin pigment can be used as a potential antitumor agent, as it exhibited a strong anticancer against SK-MEL-28 with low cytotoxicity to normal, noncancerous cells. Similar results were reported by Arun et al. [44] on HEP2 carcinoma cell. 90% of cell death reported by the HeLa was reported at 300 mg/mL of cellular induction [19]. Anti-inflammatory activity of extracted melanin from fungus against cancer cell lines has been confirmed in previous studies by Pombeiro-Sponchiado et al. [45]. Melanin pigment is highly regulated in its membrane and thus exhibits anti-inflammatory activity [46]. The melanin pigment prevents the processes, promoting or strengthening cellular contents overexpression [47]. The leaf extract of *Artemisia nilagirica* (Clarke) exhibited good anti-inflammatory activity with maximum protection and minimum hemolysis (74.63% and 25.37%) [48].

**Table 1:** Antibacterial activity against pathogenic bacteria.

Pathogenic Bacteria	Zone of inhibition in diameter (mm) of different concentrations of Melanin (μg/mL)			
	31.25	62.5	125	250
*Bacillus cereus*	13±0.07	15±0.04	18±0.02	25±0.07
*Escherichia coli*	12±0.20	15±0.04	18±0.16	21±0.12
*Staph*. *aureus*	17±0.08	20±0.02	22±0.05	22±0.09
*P*. *aeruginosa*	16±0.11	17±0.07	19±0.07	20±0.04
*K*. *pneumoniae*	5±0.04	7±0.08	9±0.09	12±0.15

Values are the average of triplicates. ± indicates standard deviation.

In addition to the anticancer study, wound healing is appropriate. Cell migration plays an important role in wound repair, and hence cell migration assay was performed to examine the wound healing ability of melanin pigment. Yet, this analysis is an inexpensive method to validate cell migration activity directly correlates with wound healing [49]. In this study, cell migration efficiency decreased with increased melanin concentration and previous studies reveal similar activity by antibiotics produced *S*. *puniceus* AS13 [31]. Hence, further studies exploring various metabolites from strain *S*. *puniceus* RHPR9 would contribute to its potential use in the pharma and food industry.

## Conclusion

Medicinal plants and their products have been used in traditional medicine for ages. They serve as a source of a wide range of bioactive molecules like antibiotic, antiviral, and antifungals. *S*. *puniceus* RHPR9 isolated from the rhizosphere of *C*. *fenestratum* produced melanin with wide applications ies. Further, this study provided a new framework to research by establishing multiple functional and characteristic activities of melanin like antibacterial, antioxidant, anticancer, anti-inflammatory, cell migration properties, etc., *in vitro* for the drug discovery patterns. Accordingly, these findings have set the background for further mechanistic studies to identify secondary metabolites of Streptomyces spp. with efficient therapeutic approach in anticancer drug discovery.
